# Cold Temperature Encoding by Cutaneous TRPA1 and TRPM8-Carrying Fibers in the Mouse

**DOI:** 10.3389/fnmol.2017.00209

**Published:** 2017-06-30

**Authors:** Zoltan Winter, Philipp Gruschwitz, Stephanie Eger, Filip Touska, Katharina Zimmermann

**Affiliations:** Department of Anesthesiology, University Hospital Erlangen, Friedrich-Alexander-University Erlangen-NürnbergErlangen, Germany

**Keywords:** cold transduction, nociceptor, thermoreceptor, thermal preference behavior, cold avoidance, C57BL/6J, 129S1/SvImJ, strain difference

## Abstract

Previous research identified TRPM8 and TRPA1 cold transducers with separate functions, one being functional in the non-noxious range and the second one being a nociceptive transducer. TRPM8-deficient mice present overt deficits in the detection of environmental cool, but not a lack of cold avoidance and TRPA1-deficient mice show clear deficits in some cold nocifensive assays. The extent of TRPA1's contribution to cold sensing *in vivo* is still unclear, because mice lacking both TRPM8 and TRPA1 (DKO) were described with unchanged cold avoidance from TRPM8^−/−^ based on a two-temperature-choice assay and by c-fos measurement. The present study was designed to differentiate how much TRPM8 alone and combined TRPA1 and TRPM8 contribute to cold sensing. We analyzed behavior in the thermal ring track assay adjusted between 30 and 5°C and found a large reduction in cold avoidance of the double knockout mice as compared to the TRPM8-deficient mice. We also revisited skin-nerve recordings from saphenous-nerve skin preparations with regard to nociceptors and thermoreceptors. We compared the frequency and characteristics of the cold responses of TRPM8-expressing and TRPM8-negative C-fiber nociceptors in C57BL/6J mice with nociceptors of TRPM8-deficient and DKO mice and found that TRPM8 enables nociceptors to encode cold temperatures with higher firing rates and larger responses with sustained, static component. In TRPM8^−/−^, C-fiber cold nociceptors were markedly reduced and appeared further reduced in DKO. Nevertheless, the remaining cold responses in both knockout strains were similar in their characteristics and they were indifferent from the TRPM8-negative cold responses found in C57BL/6J mice. TRPM8 had a comparably essential role for encoding cold in thermoreceptors and lack of TRPM8 reduced response magnitude, peak and mean firing rates and the incidence of thermoreceptors. The encoding deficits were similar in the DKO strain. Our data illustrate that lack of TRPA1 in TRPM8-deficient mice results in a disproportionately large reduction in cold avoidance behavior and also affects the incidence of cold encoding fiber types. Presumably TRPA1 compensates for lack of TRPM8 to a certain extent and both channels cooperate to cover the entire cold temperature range, making cold-temperature encoding by TRPA1—although less powerful—synergistic to TRPM8.

## Introduction

Mice, like the C57BL/6J laboratory mouse strain, show naturally a robust preference for warm over cold temperatures. Several mouse behavioral assays were used to quantify this trait. The avoidance of cold is reduced to a variable extent in mice lacking either of the transient receptor potential ion channels, TRPM8 or TRPA1, which are widely accepted as cold transduction channels in somatosensory nerves. While the function of TRPM8 is well defined, the extent of TRPA1's contribution to the cold percept is still a matter of debate. In addition, the identity of the residual cold avoidance in TRPM8-null mutants remains to be defined.

The lack of cold avoidance in TRPM8-null mice (TRPM8^−/−^) was first quantified in a two-temperature choice (2TC) assay and the phenotype is large between 25 and 15°C, but became less apparent at lower, noxious temperatures. This phenotype is robust; although it is dependent on the assay configuration (plate size and measurement time), it was identified independently across different research groups. This is in contrast to the measurement of the latency to paw withdrawal from a cold plate, where behavior of TRPM8-null mice appeared highly variable (Bautista et al., 2007; Colburn et al., 2007; Dhaka et al., 2007). Comparable to the results from the 2TC assays, measurement on a linear gradient assay adjusted between 15 and 54°C showed a larger tolerance of TRPM8^−/−^ for colder temperatures which became apparent as longer periods of exploration with little preference were mice located around 22°C, much lower than wildtype littermates (Dhaka et al., 2007).

TRPA1-null mice (TRPA1^−/−^), showed quite variable results in the paw withdrawal assay from a 10 to 0°C cold plate (Kwan et al., 2006; Karashima et al., 2009). When probed for cold reflex responses in a new test where a piece of dry ice is applied directly under the hind paw through a glass plate (Brenner et al., 2012), TRPM8^−/−^ and TRPM8-DTR-mice had a pronounced prolongation of the response, but TRPV1-DTR mice, which lack TRPA1 expression, had unchanged responses and mice lacking both TRPM8- and TRPA1-pathways (TRPV1-DTR/TRPM8-DTR mice) were found indistinct from TRPM8-DTR animals (Pogorzala et al., 2013). In addition, TRPA1^−/−^ and mice lacking TRPM8 and TRPA1 showed no altered behavior at any combination of plate temperatures in the 2TC (Knowlton et al., 2010). Results from functional Magnetic Resonance Imaging, however, illustrated that 15°C contact stimulation of the paw entailed a general reduction of the BOLD signal. This discrepancy indicates that the current mouse behavioral assays are not sensitive enough to isolate and quantify the contribution of TRPA1 to cold perception or that it's lack is well-compensated by other pathways. The reasons may lie in the very recent finding that TRPA1 acts also as heat sensor (Moparthi et al., 2014) and the complex wiring of temperature-sensing pathways via inhibitory crosstalk in the spinal cord (McCoy et al., 2013).

We have recently described a novel circular thermal gradient assay as useful tool for detailed thermal preference phenotyping (Touska et al., 2016). TRPA1^−/−^, without displaying any cold avoidance deficits, showed a significantly faster recognition of warm temperatures in the range between 15 and 40°C. TRPM8^−/−^, in contrast, displayed a large cold avoidance deficit in the circular gradient environment with low thermal resolution (0.5°C/cm). When the thermal resolution was increased alongside with the ring size (0.3°C/cm) the cold avoidance phenotype appeared reduced except for a broader distribution about the weighted preference temperature in the last 15 min bin. The compensation was found due to TRPA1, because a lack of both channels, TRPA1 and TRPM8 (DKO), dramatically increased the cold avoidance deficit to an extent similar to the phenotype of TRPM8^−/−^ observed in the small ring setup (Touska et al., 2016). These findings were in contrast to a previous study which characterized DKO cold avoidance as indifferent from TRPM8^−/−^ based on results from a 2TC assay and by measurement of c-fos expression in the spinal cord (Knowlton et al., 2010).

We revisited the DKO to obtain more insight into the exact contribution of TRPA1 to primary afferent cold detection in the mouse. We used the circular gradient device and adjusted the temperature of the ring between 5 and 30°C. We compared these results with the 15–40°C environment. In addition, we performed skin nerve recordings to search for encoding deficits in cold nociceptors and thermoreceptors in TRPM8^−/−^ and DKOs. We provide the first detailed data of firing properties and incidence of cold thermoreceptors in both strains. We also characterize the properties and incidence of cold nociceptors and compare them with TRPM8-positive- and TRPM8-negative cold nociceptors of the background C57BL/6J strain. We also show that the basic properties of both fiber types are maintained to large parts in the 129S1/SvImJ strain, which is genetically distant from the C57BL/6J mice. Our results confirm TRPM8 as unique cold transducer enabling sustained responses and high firing rates and estimate a considerably large contribution of TRPA1 to both innocuous cold and noxious cold sensing in the mouse somatosensory system.

## Methods

### Animals

For the behavioral experiments, we used adult TRPM8^−/−^ (Dhaka et al., 2007) which were backcrossed for six generation on C57BL/6J background and obtained from pairs of homozygous TRPM8^−/−^, and TRPA1^−/−^ (Kwan et al., 2006), back-crossed on 13 generations on C57BL/6J mice. From both we crossed and bred DKO and we used one common age- and sex-matched control group obtained from the DKO crossing and named C57BL/6J, because backcrossing were of the C57BL/6J strain purchased from Charles River (Sulzfeld, Germany). All mice were between 60 and 85 days; transgenic mice were genotyped according to our previously published procedures (Vetter et al., 2012, 2013). For the skin-nerve recordings of DKO shown in Figures **5**, **6** we used 22 adult mice (4 females and 17 males). For the recordings shown in Figure **4** and the recordings from TRPM8^−/−^ nociceptors, please refer to the details outlined in Vetter et al. (2013). The data underlying Figure **6** were recorded from five adult male TRPM8^−/−^ and three adult male C57BL/6J mice and include the recordings of C57BL/6J CC-fibers shown in Toro et al. (2015). Recordings from 129S1/SvImJ mice were subjected to new analysis but were all from Zimmermann et al. (2011). A-fiber nociceptors in C57BL/6J mice were new and recorded from 22 adult mice (9 females and 13 males).

### Temperature gradient assay

We utilized the large and high thermal resolution ring configuration of our previously introduced circular temperature gradient assay (Touska et al., 2016). We quantified cold avoidance in TRPM8^−/−^ and DKO in the temperature range from 30 to 5°C. The data were from the same mice previously measured in the 15–40°C environment (Touska et al., 2016). During these experiments, all mice were adapted to the equipment on day 1 with the ring adjusted to room temperature for 30 min. Mice were measured for 60 min on day 2 using 15–40°C and on day 3 using 5–30°C. To achieve a symmetric gradient with a midpoint temperature of 17.5°C, we air-conditioned the room to 17–18°C, otherwise the room was heated to 26°C using a convector heater. Behavior was videotaped with a CCD-camera and analyzed with our custom-designed software described and validated in Touska et al. (2016). The protocol for *in-vivo* experiments in animals was reviewed by the local animal ethics committee (University of Erlangen) and approved by the local district government.

### Isolated skin nerve preparation and single-fiber recordings

We performed electrophysiological recordings as previously described (Zimmermann et al., 2009, 2011; Vetter et al., 2013; Toro et al., 2015). Briefly, single-fiber activity was recorded from teased fibers via platinum or gold wire electrodes in an adjacent chamber overlaid with paraffin oil. Receptive fields were isolated from the surrounding fluid by means of a teflon ring. Cold sensitivity was tested by superfusion of the receptive field with precooled synthetic interstitial fluid (SIF). Well-defined cold stimuli were realized with a custom-designed counter-current temperature exchange system and they reached in nociceptors from bath temperature (30–32°C) to 8.3 ± 2.8°C and in thermoreceptors from bath temperature (33–35°C) to 7.3 ± 2.4°C in 60 s. *Cold nociceptors* were identified by searching mechanosensitive receptive fields with a glass rod and isolation of the receptive field with the teflon ring. Specifically, we recorded populations of C-fibers from DKO, TRPM8^−/−^ and A- and C-fibers from C57BL/6J. Fibers from several previous studies were analyzed retrospectively to specifically characterize the properties of TRPM8+ and TRPM8− cold nociceptors in the C57BL/6J and the 129S1/SvImJ mouse strains. *Thermoreceptors* were identified by splitting nerve bundles until C-fiber activity was noted and at least one and maximal five mechanosensitive receptive fields could be identified on the skin. This served to adjust the amplification range for each and every split to a level that undoubtedly detects C-fiber activity with a high enough signal-to-noise ratio. This is crucial, because the thermoreceptors stem from the smallest diameter dorsal root ganglia neurons and are expected to require close contact with the recording electrode. Subsequently, to recognize cold sensitive spots, a small ice cube (1 cm^3^) was slowly moved very closely over the corium side of the skin-nerve preparation without touching the receptive areas of the skin. Thermoreceptor activity can be recognized by immediate onset brisk firing at a high rate that ceases shortly after the ice cube is taken away from the respective area. To account for a faster equilibration of the bath temperature, we increased the flow and the bath temperature to 33–35°C. The respective area is then isolated with a teflon ring and the receptive field is subjected to controlled thermal stimulation (Zimmermann et al., 2009). Adjustments of the ring location are made if necessary.

### Statistical analysis

Comparisons between two groups were performed using *T*-test for paired or unpaired samples, respectively; for more than two groups one-way ANOVA' planned comparison with Fisher LSD *post-hoc* test were computed using IBM SPSS Statistics version 21. Differences were considered significant at *p* < 0.05 and are marked by asterisks, hashtags, or dollar signs as indicated in figure legends. For skin nerve data we used the Grubbs's outlier test to identify outliers. Outliers were marked in Figures **4**, **5** with stars. The outlier values were not included in the calculation of the mean and quartiles and were also removed for the statistical calculation. Error bars in figures are displayed as *SEM* or *SD*, as indicated in figure legends. In figures “^***^” symbolizes *p* < 0.001, “^**^” signifies *p* < 0.01 and “^*^” represents *p* < 0.05.

## Results

### Mice lacking TRPA1 and TRPM8 have larger deficits in avoidance of noxious and innocuous cold than TRPM8-deficient mice

In our previous study, we measured the thermal preference behavior of TRPM8^−/−^ and DKO in a thermal gradient assay equilibrated between 15 and 40°C. We found that TRPM8-deficient mice show a remarkable lack of cold avoidance in the assay configuration with low thermal resolution and steep gradient (0.5°C/cm; 3.6°C between individual fields), but nevertheless they still do recognize warmer zones as preferable to colder areas, but they require longer to locate to the warmer zones. Remarkably, in an environment with a shallower gradient and increased thermal resolution (0.3°C/cm, 2.3°C between fields), the lack of TRPM8 is well-compensated and the cold avoidance deficit is no longer apparent. Here, the only difference to the wildtype is a broader range of preferred temperatures visible in a less negatively skewed distribution in the last 15 min of the acquisition (Touska et al., 2016). Remarkably, additional lack of TRPA1 created a similarly large lack of cold avoidance in the DKO as previously recognized in the TRPM8^−/−^ strain in the smaller ring with the steep gradient. To compare these data with data acquired in a 5–30°C environment of the large ring with the shallow gradient, we calculated a cumulative response function for the early, explorative behavior in the first half hour (Figure 1A) and the late, thermal preference behavior (Figure 1B) acquired in the last 15 min. Remarkably, in the 15–40°C environment, the DKO show random exploratory behavior below 32°C devoid of any cold avoidance (*p* > 0.2), but intact avoidance of the warmer fields >34°C (*p* = 0.03, *p* = 0.000001, and *p* = 0.00004). In contrast, the TRPM8^−/−^ are indifferent from wildtype. In this temperature range, with a minimum temperature of 15°C, and with this thermal resolution, obviously, presence of either TRPA1 and TRPM8 is sufficient to produce acute cold avoidance, because lack of each single channel does not make any cold avoidance deficits apparent—in the case of TRPA1, mice are even more sensitive to cold than control mice (at 32°C, Figure 1A and Touska et al., 2016). Cold avoidance vanishes only when both channels are deficient. With longer exposure, i.e., in the last 15 min of the 1 h observation, in the DKO, a third, probably slow onset cold detection mechanism, primary afferent or central, unfolds and a considerable amount of cold avoidance becomes apparent although the DKO still have an outstandingly large tolerance for colder ring areas; they spend significantly less time than C57BL/6J between 26 and 34°C and, when compared to TRPM8^−/−^, this concerns the entire temperature range between 15 and 34°C (Figure 1B). When we compared the early and late behaviors, as illustrated in Figures 1A,B, we found it to be different in all strains for the temperatures below 28°. These findings underline the assumption that time is a significant factor in a temperature gradient setup (Table 1) and that the early and late bins should be regarded separately.

**Figure 1:** Cumulative response functions of preferred temperature zones measured with gradients of 15–40°C **(A,B)** and 5–30°C **(C,D)**. X-axis represents the temperature between each of the 12 zones, Y-axis indicates percent time each group has spent above the indicated zone temperature. Panels **(A,C)** refer to min 1–30 (exploratory behavior) and **(B,D)** refer to late behavior in min 46–60 (thermal preference selection). The dashed gray line represents expected random zone coverage estimated from the surface size of each thermal section, i.e., >16 or 6°C: 92%; >18 or 8°C: 83%; >21 or 11°C: 75%; >23 or 13°C: 67%; >25 or 15°C: 58%; >28 or 18°C: 50%; >30 or 20°C: 42%; >32 or 22°C: 33%; >34 or 24°C: 25%; >37 or 27°C: 17%, and >39 or 29°C: 8%. Note, that increasing thermal selection behavior becomes apparent in the last 15 min of both experiments. C57BL/6J (*n* = 20): black triangles, TRPM8^−/−^ (*n* = 19): cyan triangles, TRPA1^−/−^ [*n* = 20 **(A,B)** and 16 **(C,D)**]: red diamonds, DKO (*n* = 20) blue circles. Asterisks in black and cyan indicate significant differences for *p* < 0.05 (ANOVA) between DKO and C57BL/6J and DKO and TRPM8^−/−^, respectively. Black # and $: significant differences for *p* < 0.05 (ANOVA) between TRPM8^−/−^ and TRPA1^−/−^ and C57BL/6J, respectively. Whiskers represent S.E.M. Note that Table 1 illustrates *p*-values for early and late behavior of each strain.

**Table 1:** Comparison of early and late behavior in the thermal ring track.

	**C57BL6J**	**TRPA1**	**TRPM8**	**DKO**
**15–40°C**				
16.1°C	0.0001083	0.0001813	0.0000002	0.0029062
18.4°C	0.0000068	0.0002176	0.0000006	0.0001862
20.7°C	0.0000013	0.0005667	0.0000004	0.0000320
23.0°C	0.0000026	0.0001971	0.0000003	0.0001017
25.2°C	0.0000002	0.0000908	0.0000004	0.0000142
27.5°C	0.0000001	0.0001455	0.0000001	0.0007774
29.8°C	0.0000002	0.0000530	0.0005536	0.0113807
32.0°C	0.0000001	0.0000244	0.0009478	n.s.
34.3°C	0.0083921	n.s	0.0153580	n.s.
36.6°C	n.s	0.0053769	0.0031597	n.s.
38.9°C	0.0000124	0.0188530	0.0000009	0.0000134
**5–30°C**				
6.1°C	0.0000012	0.0000717	0.0000580	0.0000556
8.4°C	0.0000002	0.0000072	0.0000297	0.0000841
10.7°C	0.0000004	0.0000202	0.0000063	0.0000880
13.0°C	0.0000003	0.0000528	0.0000044	0.0002339
15.2°C	0.0000002	0.0000302	0.0000046	0.0001636
17.5°C	0.0000006	0.0000629	0.0000179	0.0000525
19.8°C	0.0000001	0.0002255	0.0000014	0.0000049
22.0°C	0.0000002	0.0001433	0.0000004	0.0000008
24.3°C	0.0000000	0.0001887	0.0000001	0.0000041
26.6°C	0.0000000	0.0000887	0.0000302	0.0000779
28.9°C	0.0000002	0.0000005	0.0066261	0.0096410

*P-values were calculated for all data points of the cumulative preference graph for each strain as shown in Figure 1 (paired t-test) and yield time as an important influential factor in this experiment*.

We next analyzed the behavior of the same groups of mice in the circular running track with temperatures between 5 and 30°C (Figures 1C,D). Remarkably, exploratory behavior was guided by cold avoidance in all strains. Yet, the DKO showed least cold avoidance and were significantly different from TRPM8^−/−^ at all temperatures (*p* < 0.05, ANOVA), except for 30°C (*p* = 0.092, ANOVA). When compared to the wildtype littermates, TRPM8^−/−^ showed less cold avoidance only >24°C and the cumulative response function for TRPA1^−/−^ seemed shifted to higher temperatures, but this was significant only for 30°C (*p* < 0.0001, ANOVA; Figure 1C). In the last 15 min of the 1 h observation, the DKO showed a large tolerance for colder ring areas and they occupied all fields ≤29°C longer than TRPM8 or control mice (Figure 1D). For all temperatures ≤24°C TRPM8^−/−^ were again indifferent to control mice but they showed—similar to the 15–40°C environment—a broader range of thermal preference spending significantly less time at temperatures above 27° (Figure 1D). Comparison of the early and late behaviors was different in all strains with higher levels of significance than observed for the 15–40°C environment (Figures 1C,D and Table 1, bottom columns).

The preference temperature time course shown in Figure 2A further illustrates the large differences in the cold avoidance phenotypes of TRPM8^−/−^ and DKO. Virtually all timepoints of the timecourse of DKO locate to significantly lower weighted preferred temperatures in comparison to both TRPM8^−/−^ and wildtype (Figure 2A). In addition the DKO had significantly larger *SD*, even in the last 15 min of the measurement, than wildtype and TRPM8^−/−^, which is indicative of a more erratic behavior and a larger tolerance for the lower temperatures (Figure 2A and Table 1). Again, similar to the 15–40°C environment, TRPA1^−/−^ appeared to be more sensitive to cold and seemed to recognize the warmer areas faster (not shown in Figure, compare parameters listed in Table 2). In the final 15 min of the experiment, TRPM8^−/−^ located at 1.2°C lower than wildtype (*p* = 0.2, ANOVA, Table 2), but only the DKO displayed a significant reduction of preferred temperature choosing 4.3°C lower than wildtype and 3.1°C lower than TRPM8^−/−^ (*p* = 0.0001, ANOVA, Table 2).

**Figure 2:** Characterization of cold avoidance behavior in DKO in the 5–30°C gradient. **(A)** Preference temperature time course in minute resolution illustrates a significant segregation of weighted preferred temperatures of DKO (*n* = 20, dark blue) and TRPM8^−/−^ (*n* = 19, cyan with white whiskers) and C57BL/6J mice (*n* = 20, gray). Note that DKO migrate to warmer zones, but have a higher SD than any other of the strains illustrating a broader tolerance for cold temperatures. Data are 3pt averaged. Error bars are *SD* (2nd moment). **(B)** Zone preference histograms of exploratory (1–15 min, bottom) and thermal preference behavior (46–60 min, top) of C57BL/6J (gray), TRPM8^−/−^ (cyan), and DKO (blue). Exploratory behavior (bottom) illustrates that DKO avoid colder floor temperatures less than TRPM8^−/−^ and all other strains. The deficit in cold avoidance of DKO becomes larger at the end of the observation time and leads to occupation of cooler floor temperatures (top). Error bars indicate S.E.M. **(C,D)** Time courses of thermal selection. Percent time spent **(C)** >24.3°C and, **(D)** >28.8°C calculated in 1 min resolution (average of 60 values per min) and subjected to 3 pt averaging. **(C)** Cold avoidance deficits of DKO become apparent in comparison to C57BL/6J and TRPM8^−/−^, but DKO still prefer warmer areas and require more time to locate there (dashed line: 25.0% random probability). **(D)** Using the 30°C field as discriminator, makes graded phenotypic differences between all three strains apparent (dashed line: 8.3% random probability). Error bars indicate S.E.M. Asterisks in black and cyan indicate significant differences for *p* < 0.05 (ANOVA) between DKO and C57BL/6J and DKO and TRPM8^−/−^, respectively. Black #: significant differences for *p* < 0.05 (ANOVA) between TRPM8^−/−^ and C57BL/6J.

**Table 2:** Comparison of the strains in the 5–30°C assay.

**Bins**	**Strains**	**descriptors of distribution**		
		**Mean (°C)** ± ***SD***	***SD***	**Skew**
1–15 min	WT (C57Bl/6J)	21.82 ± 1.9	6.96	−0.61
	TRPA1^−/−^	23.33 ± 2.7	6.70	−0.95
	TRPM8^−/−^	20.24 ± 2.0	7.01	−0.45
	DKO	18.44 ± 2.0	7.46	−0.14
15–30 min	WT (C57Bl/6J)	26.12 ± 0.7	5.86	−1.74
	TRPA1^−/−^	27.60 ± 3.6	4.73	−2.26
	TRPM8^−/−^	24.54 ± 3.1	6.24	−1.27
	DKO	21.38 ± 3.5	7.45	−0.62
30–45 min	WT (C57Bl/6J)	28.96 ± 0.6	4.44	−2.94
	TRPA1^−/−^	28.72 ± 2.2	2.96	−3.20
	TRPM8^−/−^	26.81 ± 3.2	4.96	−2.25
	DKO	23.52 ± 4.1	7.08	−1.11
45–60 min	WT (C57Bl/6J)	28.68 ± 2.3	3.73	−3.57
	TRPA1^−/−^	29.31 ± 1.2	2.20	−3.93
	TRPM8^−/−^	27.46 ± 2.2	4.08	−2.78
	DKO	24.37 ± 4.1	6.85	−1.37

*Values of preference temperature, SD, and Skew in the circular running track equilibrated between 5 and 30°C. The skew in the 5–30°C environment is negative and extends a tail to the left. TRPM8^−/−^ and DKO have a broader distribution extended to lower temperatures which results in a less negative skew. The double knockouts have the least left-skew distributions in all bins. This appears alongside with lower preferred temperatures. Compare Touska et al. (2016) for the respective values in the 15–40°C gradient*.

A more detailed view of the evolution of the cold avoidance phenotype over time provides the histogram chart of the first and last 15 min bins. It becomes apparent that in the first 15 min DKO avoided the colder zones ≤15°C much less than both wildtype and TRPM8^−/−^ (Figure 2B, lower panel). In the last bin of measurement time, the phenotype became more obvious to include all ring areas ≤24°C. Much in contrast, both TRPA1^−/−^ (not shown) and TRPM8^−/−^ showed adequate cold avoidance for these ring zones and were insignificantly different from wildtype. The lack of TRPM8 distinctively affected only temperatures above 24°C, where the TRPM8^−/−^ spent less time on the 30°C field and located instead rather between 25 and 28°C. Of all strains, the DKO spent the least time on the 30°C field (Figure 2B, upper panel). The temperatures of the largest phenotypic difference between TRPM8^−/−^ and wildtype was the range of 28–30°C and for the DKO and wildtype the range reached from 24–30°C. Therefore, we calculated time courses of thermal selection for these two surface sections which cover the warmest 25 and 8% of the ring area. For both time courses, DKO and TRPM8^−/−^ are significantly segregated at almost all time points, while the TRPM8^−/−^ displayed its largest differences to the wildtype for discrimination of 28°C. In numbers, the C57BL/6J mice required 16 min to spend at least 2/3rd or more of their time >24°C, the TRPM8^−/−^ required 22 min while the DKO never showed such a large selection for the temperature >24°C. The differences between genotypes became larger when regarded for the temperature >28°C, where C57BL/6J mice required 34 min to spend 2/3rd or more of their time and both TRPM8^−/−^ and DKO never showed such a large preference (Figures 2C,D).

Last but not least, we analyzed the general activity or locomotion of the strains in the ring assay as amount of zone transitions in the warm and cold thirds (Figure 3). For the cold third this includes the large field that is required for automated analysis (Touska et al., 2016) which is why counts include transitions between five fields, while for the warm third the data includes transitions between six fields (see sketches in Figure 3). We therefore compared transitions in cold and warm thirds between strains and between the 15–40°C (Figures 3A,B) and 5–30°C environments (Figures 3C,D). In all strains, and in both environments, the number of transitions was higher in the first half as compared to the second half of the measurement. In the 5–30°C environment, remarkably, TRPA1^−/−^ had the least number of zone transitions in the cold third and avoided entering the cold areas in the second half of the experiment (*p* < 0.0001, 41.7 early and 2.5 late transitions in the cold third; Figure 3C). While TRPM8^−/−^ (73.1 early and 18.5 late transitions in the cold third) were remarkably similar to C57BL/6J (66.5 early and 19.5 late), DKO showed more than twice as many zone transitions (154.3 early and 90.5 late) and, in contrast to all other strains, the cold avoidance was not much increased in the second half hour (*p* < 0.001, paired *T*-test; Figure 3C). With respect to the zones >22°C, again DKO showed the largest number of transitions in both the early and late halves (early: *p* < 0.0001 vs. TRPA1 and *p* = 0.02 vs. TRPM8^−/−^; late: *p* < 0.001 vs. TRPA1, *p* = 0.001 vs. TRPM8, and *p* = 0.047 vs. C57BL/6J, ANOVA) while TRPA1^−/−^ moved significantly less than C57BL/6J (*p* = 0.048 ANOVA; Figure 3D). When comparing the 15–40°C and 5–30°C environments, we found that the DKO behaved indifferent in the respective cold thirds, but different in the warm thirds for both early (cold: *p* = 0.8 and warm: 0.002) and late (cold: *p* = 0.3 and warm: 0.009). Remarkably, TRPA1^−/−^ had significantly less zone transitions in the 5°C cold third as compared to the 15°C cold third for both early (*p* = 0.0004) and late (*p* = 0.02, Student's *t*-test; Figures 3A,C).

**Figure 3:** Locomotor activity in warm and cold ring thirds. Locomotor activity is calculated as the number of individual zone transitions and illustrated as bar chart for each strain and early (1–30 min, dark colors) and late (31–60 min, light colors) time bins. Sketches illustrate that zone transitions are calculated separately for **(A,B)** the 15–40°C environment with **(A)** the cold ring third <23°C and **(B)** the warm ring third (>32°C) and **(C,D)** the 5–30°C environment with **(C)** the cold ring third <13°C and **(D)** the warm ring third (>22°C). Note that all strains show fewer transitions in the 2nd 30 min in all conditions. Note that TRPA1^−/−^ show strong cold avoidance in **(C)** and the least transitions in the cold and completely avoid cold fields in the 2nd 30 min. DKO show almost three times as many transitions as C57BL/6J or TRPM8^−/−^ in the cold **(C)** and they exhibit the highest number of zone transitions in the warm third **(D)**. Asterisks and hashtags refer to ANOVA *p* < 0.05 and compare early and late values, respectively. *N* = 16–20 mice per strain. For details see text.

These large behavioral phenotypic differences of the DKO made apparent that lack of TRPA1 may cause larger deficits in primary afferent cold detection than previously assumed. To define the exact primary afferent electrophysiological correlates contributed by TRPA1 and TRPM8, we quantified cold responses of cold-sensitive fiber types in the mouse saphenous nerve for TRPM8-positive and TRPM8-negative fibers of C57BL/6J, TRPM8^−/−^, and DKO.

### TRPM8 increases cold responses and static discharge of mechanocold C-fiber nociceptors

We first assessed cold nociceptors (C-mechano-cold, CMC, and C-mechano-cold-heat, CMCH) and revisited our previous sampling studies performed mainly in the background C57BL/6J strain, but also in littermates of TRPM8^−/−^ (Vetter et al., 2013) where a distinction was made between TRPM8-positive and TRPM8-negative cold nociceptors based on pharmacological evidence. In the respective studies, all fibers were searched randomly using a glassrod and the effects of menthol 50 or 500 μM, camphor 2 mM and XE991 10 and 100 μM on the cold response were quantified after previous superfusion of the receptive field for 4–5 min with these compounds at bath temperature. All named compounds sensitize to cold only in presence of a functional TRPM8 receptor (Zimmermann et al., 2011; Vetter et al., 2013; Toro et al., 2015). One hundred and eight C-mechano fibers were included and subjected to a new analysis where the cold sensitive fibers (>3 spikes per 60 s cold stimulus) were segregated into the two populations. In contrast to our previous publications, we classified fibers now as CMC if they had zero spikes during a heat ramp and as CMCH if they had at least one spike during the heat stimulation, discharged close to or at ramp's peak, at least >44°C. In CMC fibers, a burst in the middle of the heat ramp around 40–44°C is interpreted as paradoxic heat response. With these criteria, 19 CMC and 29 CMCH were identified and, thereof 15 CMC and 3 CMCH were positive for a functional TRPM8. When we characterized the properties of the cold responses in these four groups, we found that TRPM8-positive CMC fibers (*n* = 26) generate 2.2-fold larger responses and 2-fold higher peak firing rates than TRPM8 negative (*n* = 4) CMCs (see Table 3; *p* > 0.05, Student's *t*-test). In CMCH-fibers, TRPM8 caused a 3.5-fold larger response and increased the peak discharge by 1.2-fold (*p* < 0.001 Student's *t*-test; compare Table 3). Irrespective of the fiber type, the difference a functional TRPM8 makes to a cold nociceptor's response reflects in an almost 4-fold difference in response magnitude (24.7 ± 17.5 vs. 6.4 ± 3.5, *p* < 0.001, Student's *t*-test, *n* = 30 each, Figures 4A,B) and leads to higher peak (3.4 ± 2.8 vs. 2.0 ± 3.5, *p* = 0.03; Figure 4C) and mean discharge rates (0.8 ± 0.6 vs. 0.5 ± 0.4, *p* = 0.003). The presence of TRPM8 has also unique effects on the shape of the response as it enables the fibers to produce a sustained static response with much less adaptation in contrast to TRPM8-negative fibers. With TRPM8 present, more than 84% of the response is discharged within seconds 16–60 of the stimulus, where the temperature has already reached below 12°C and is only changing at a very slow rate. The static response is reduced to 55% in absence of TRPM8 (*p* = 0.00005, Student's *t*-test, *n* = 30 each, Figures 4A,D). Interestingly, in the C57BL/6J strain, TRPM8-positive nociceptors have 5°C lower threshold temperatures and started to discharge when the temperature reaches 18.4°C ± 4.7, while the TRPM8-negative nociceptors activated already at 23.5°C ± 5.7 (*p* = 0.0001, Student's *t*-test; Figure 4E).

**Table 3:** Properties and occurrence of cold nociceptor subtypes in mice of the strains C57BL/6J, 129S1/SvImJ, TRPM8^−/−^, and DKO.

**Strain/C-fibers**	**Cold sens. C-fibers**	**Fiber type**	**Relative frequency (*n*) and TRPM8 pharmacology (+/−)**			**Number of action potentials per 60 s cold stimulus**	**Static response as % of entire response**	**Peak DC (1/s)**	**Mean DC (1/s)**	**Thresh. temp. (°C)**	**Conduction velocity (m/s)**	**von Frey threshold (mN)**
										**Mean (min/max)**	**Mean (min/max)**	**Median (min/max)**
C57BL/6J *n* = 108	48 (44%)	CMC	19(40%)	+	15(79%)	24.9 ± 18.4^a^(*n* = 26)	84.0 ± 11.3^a^	3.5 ± 2.7^a^	0.8 ± 0.6^a^	18.5 ± 4.6 (11.1/27.4)^a^	0.43 ± 0.10 (0.22/0.63)^a^	4(1/45.3)^a^
				−	4(21%)	11.5 ± 9.0(*n* = 4)	46.8 ± 20.8	1.7 ± 1.0	0.6 ± 2.3	23.6 ± 4.9 (17.7/27.6)	0.53 ± 0.25 (0.36/0.90)	5 (2/22.4)
		CMCH	29(60%)	+	3(10%)	22.7 ± 8.1	83.3 ± 23.6	2.4 ± 1.1	0.8 ± 0.3	17.4 ± 4.7 (14.3/15.1)	0.58 ± 0.27 (0.42/0.90)	4 (2.8/8)
				−	26(90%)	6.6 ± 3.6	54.5 ± 40.3	1.9 ± 3.5	0.45 ± 0.4	23.5 ± 5.6(30.9/8.7)	0.41 ± 0.10(0.24/0.58)	8(1.4/128)
		CMC and CMCH		+	18(37%)	24.7 ± 17.5^a^(*n* = 30)	84.6 ± 11.8^a^	3.4 ± 2.8^a^	0.8 ± 0.6^a^	18.4 ± 4.7^a^	0.45 ± 0.13 (0.22/0.90)^a^	4 (1/45.3)^a^
		CMC and CMCH		−	30(63%)	6.4 ± 3.5(*n* = 30)	54.5 ± 41.1^a^	2.0 ± 3.5	0.5 ± 0.4	23.5 ± 5.7	0.43 ± 0.13 (0.24/0.90)	8 (1.4/128)
129S1/SvImJ *n* = 55	22 (40%)	CMC	14(64%)	+	8(57%)	33.1 ± 29.3	83.1 ± 12.1	4.0 ± 2.5	1.0 ± 0.6	25.5 ± 3.8 (18.2/31.0)	0.50 ± 0.20 (0.28/0.78)	4.85 (1/16)
				−	6(43%)	5.8 ± 2.0	81.0 ± 26.0	1.5 ± 1.1	0.5 ± 0.4	19.9 ± 5.3 (13.5/26.3)	0.31 ± 0.06 (0.24/0.43)	4.85 (2.8/8)
		CMCH	8(36%)	+	–	–	–	–	–	–	–	–
				−	8(100%)	7.6 ± 8.5	59.5 ± 40.1	1.4 ± 1.8	0.5 ± 0.5	20.2 ± 6.7 (5.1/25.3)	0.32 ± 0.12 (0.23/0.47)	6.85 (1/16)
		CMC and CMCH		−	14(64%)	6.9 ± 6.4	68.6 ± 35.3	1.5 ± 1.5	0.5 ± 0.5	20.1 ± 5.9 (5.1/26.3)	0.32 ± 0.09 (0.20/0.47)	5.7 (1/16)
TRPM8^−/−^*n* = 54	16 (30%)	CMC and CMCH	1 (6%); 15 (94%)	–	–	7.6 ± 4.1	56.2 ± 25.0	1.9 ± 0.8	0.5 ± 0.3	23.7 ± 5.5 (9.0/30.1)	0.42 ± 0.09 (0.29/0.59)	5.7 (2/16)
TRPM8^−/−^*n* = 7	Mechanosensitive dynamic cold nociceptors^b^					26.4 ± 10.4	23.2 ± 18.2	6.6 ± 4.8	2.7 ± 2.0	32.0 ± 2.2 (27.6/34.1)	0.42 ± 0.06 (0.34/0.47)	7.7 (2.8/64)
DKO *n* = 38	6 (16%)	CMC and CMCH	3 and 3	–	–	10.5 ± 9.8^b^(*n* = 13)	63.0 ± 13.7^b^	2.6 ± 3.6^b^	0.5 ± 0.5^b^	23.8 ± 7.4 (6.4/30.1)^b^	0.42 ± 0.1 (0.28/0.57)^b^	8 (2.8/32)^b^

*Part of the recordings were from previous sampling studies and subjected to new grouping and analysis (Zimmermann et al., 2011; Vetter et al., 2013; Toro et al., 2015). In C57BL/6J, 108 fibers were included from unbiased sampling studies*.

a *The values from CMC fibers were calculated with inclusion of additional CMC fibers from a biased search: the occurrence of fibers subtypes was calculated for the unbiased sample and the properties refer to the entire group (n = 26)*.

b *In TRPM8^−/−^, additional fibers were identified using an ice cube as search stimulus (n = 7). Cold-insensitive fibers which develop cold-sensitivity after stimulation with TRPM8-agonists exist, but were not considered here. All values are mean ± SD*.

**Figure 4:** Cold response characteristics of TRPM8-positive and TRPM8-negative C57BL/6J mouse saphenous-nerve cold nociceptors. Distinction was based on TRPM8 pharmacology (see text) and includes CMC and CMCH types. **(A)** Averaged histogram summarizing the cold responses of all TRPM8-positive (green, *n* = 30) and TRPM8-negative (gray, *n* = 30) cold nociceptors in bins of 2s. Adjacent data points were subjected to 3pt averaging. **(B–E)** Quantification of parameters illustrates TRPM8-positive cold nociceptor responses as **(B)** larger in response magnitude counted as action potentials per 60s cold stimulus (*p* < 0.0001), **(C)** higher in peak firing frequency (*p* = 0.0001) **(D)** able to produce static, sustained responses quantified as fraction of the action potentials discharged during the constant cold stimulus (16–60 s) (*p* < 0.0001) and, **(E)** with lower threshold temperatures (*p* = 0.0002). All values are given in Table 3. Asterisks refer to Student's *t*-test. Boxes illustrate median and upper and lower quartiles. Outliers are marked with stars; one outlier in **(C)** was out of range (value 18.3); outliers were not included in calculation of mean and quartiles.

We compared the basic fiber types and their encoding characteristics to the 129S1/SvImJ mouse strain, because we wanted to know how well they were maintained across inbred strains. Both strains are evolutionary distant and belong to different groups, the Castle's mice and the C57/58 group, of the mouse family tree (Petkov et al., 2004). This or other 129-related strains are frequently used as donor strain for the generation of transgenic mice used in studies of the sensory system, including TRP-channel knockouts and backcrossing over variable generations involves a variable mixture of the genomes of both strains. In the past, assumptions about primary afferent differences in these strains were discussed as possible influence on the lack of a warm-sensing phenotype of transgenic mice lacking TRPV3 (Huang et al., 2011). The respective parameters of these fiber types for these two strains are compared in Table 3. In these strains the overall amount of cold nociceptors in the two samples was rather similar and added to 44% in C57BL/6J and 40% in 129S1/SvImJ. Interestingly, the occurrence of the fiber types CMC and CMCH was inverse, although functional TRPM8 was present in a comparable fraction of cold-sensitive fibers (*p* > 0.05, Chi-Square-test); remarkably, in the 129S1/SvImJ strain, TRPM8-positive nociceptors had almost 6°C higher threshold temperatures and started to fire at 25.5°C ± 3.8 (*n* = 8) than the TRPM8-negative nociceptors which had thresholds at 19.9°C ± 5.3 (*n* = 6, *p* = 0.04, Student's *t*-test; Table 3) which is also inverse to the C57BL/6J strain. Other parameters, such as the magnitude of the response and peak discharge rates were insignificantly different between both strains (*p* = 0.23 and *p* = 0.53, Student's *t*-test, Table 3).

### Lack of TRPM8 causes distinct encoding deficits in mechanocold C-fiber nociceptors

In two previous sampling studies conducted in TRPM8-deficient mice, which were both guided by a mechanical search stimulus, we recorded from 54 mechanosensitive C-fibers (Vetter et al., 2013) of which 16 were found to be cold sensitive. Virtually all of these fibers were CMCH and the magnitude, mean and peak discharge and the activation threshold temperature of the cold response in these fibers was indifferent from the cold response pattern of the TRPM8-agonist insensitive C57BL/6J-based group (*p* > 0.5, Student's *t*-test, Table 3, Figures 5A–E). In addition, we searched for cold sensitivity in the knockouts by slowly passing an ice cube over the skin—a search stimulus we use to identify mechanoinsensitive cold receptors as described in detail in Section Methods (Zimmermann et al., 2011). In TRPM8^−/−^ we were able to identify another population of mechanosensitive fibers with larger cold responses than the CMCH. Their response pattern was characterized by a high threshold temperature around 30°C and a vivid, dynamic cold response. Remarkably, these cold responses had a comparable magnitude as the TRPM8+ cold nociceptors in the wildtype (*p* = 0.8, Student's *t*-test, *n* = 7), but higher peak firing rates (*p* = 0.02, Student's *t*-test). In addition the static response was reduced to as much as 23% as compared to the TRPM8+ cold nociceptors (*p* < 0.001, Student's *t*-test, Table 3, Figures 5A–E. We located additional four receptive areas where at least two fibers responded vividly to cold in a similar dynamic pattern as observed with the seven single receptive fields. These fibers could not be separated to single fiber level and were therefore not included in the analysis, but they further illustrate that this type of cold response appears in relative abundance in the TRPM8^−/−^.

**Figure 5:** Cold response characteristics and relative frequency of mouse saphenous-nerve cold nociceptors in TRPM8^−/−^ and DKO. **(A)** Averaged histogram summarizing the cold responses of two populations of TRPM8-deficient cold nociceptors (dynamic, low threshold type, pink, *n* = 7 and regular type, cyan, *n* = 16) and cold nociceptors of DKO (blue, *n* = 13) cold nociceptors in bins of 2 s. Adjacent data points were subjected to 3 pt averaging. **(B–E)** Quantification of parameters illustrating **(B)** response magnitude counted as action potentials per 60 s cold stimulus, **(C)** peak firing frequency, **(D)** static response quantified as fraction of the action potentials discharged during the constant cold stimulus (16–60 s) and, **(E)** threshold temperature of activation. TRPM8^−/−^ and DKO cold nociceptor types produce cold responses with similar properties as the TRPM8-negative cold nociceptors displayed in Figure 4, but are different in all characteristics from the dynamic, low threshold TRPM8^−/−^ type (*p* < 0.008, ANOVA). **(F)** The relative frequency of regular cold nociceptors in a random sample of fibers searched by mechanical stimulation is reduced in TRPM8^−/−^ (*n* = 16 in 54) and DKO (*n* = 6 in 38) as compared to C57BL/6J (*n* = 18 TRPM8-positive and *n* = 30 TRPM8-negative cold nociceptors in 108). All values are given in Table 3. Asterisks refer to ANOVA. Boxes illustrate mean and upper and lower quartiles. Outliers are marked with stars in **(B–D)** and were not included in calculation of mean and quartiles.

### Lack of TRPM8 and TRPA1 reduces the relative frequency of mechanocold nociceptors

We performed a new sampling study guided by a mechanical search stimulus in the DKO. We recorded from 38 mechanosensitive C-fibers of 15 DKO mice. In this sample, we identified six cold sensitive fibers (see Table 3), which is about half as many as we found in TRPM8^−/−^ (Figure 5F). We also encountered 11 receptive fields were more than one fiber responded to the thermal stimulation and four of these multi-fiber recordings discharged in response to cold. Because these fibers could not be separated to single fiber level they were not included in the analysis of the cold response properties shown in Figures 5A–E. In additional eight preparations from seven mice, we used ice cubes and located additional eight receptive fields with cold sensitivity. However in none of them, we found responses similar to the properties of the mechanosensitive dynamic cold nociceptors identified in TRPM8^−/−^ and shown in Figure 5A. All cold nociceptors in DKO, except one, had low von Frey thresholds and belonged to the group of multimodal cold nociceptors. Table 3 illustrates the properties of these fibers, which were indifferent in all characteristics (response magnitude, peak discharge, and static response, *p* > 0.3) from the regular cold nociceptors identified in TRPM8^−/−^. Apparently a considerable amount of cold nociceptors remains active in DKO and produces remarkable responses although they are increasingly difficult to find.

### TRPM8 is the essential cold transducer in unimodal cold receptors

In the mouse, unimodal cold receptors were first characterized in the cornea to encode constant temperatures around 34°C with continuous, graded impulse activity and small temperature reductions with rapidly accelerating impulse activity. Corneal cold thermoreceptors are sensitive to menthol and virtually absent in the TRPM8-deficient mice (Parra et al., 2010). Depending on the subtype, they exhibit cooling thresholds around 32 or 28° and silence at 23 or 17°C, respectively (Gonzalez-Gonzalez et al., 2017). We first characterized a similar fiber type in skin-nerve preparations of 129S1/SvImJ mice (Zimmermann et al., 2011), albeit with a dynamic range that includes noxious temperatures. In the C57BL/6J strain, when compared to TRPM8-positive cold nociceptors, unimodal cold receptors have 16-fold larger responses, 18-fold higher peak, and 23-fold higher average firing rates (Figure 6A, Tables 3, 4). These properties are similar to the 129S1/SvImJ strain (Table 4). In the skin CC-fibers cover a large dynamic range with thresholds between 37 and 15°C and impulse activity encoding noxious temperatures below 10°C. Only a small fraction CC-fibers showed silencing above 17°C as it is regularly observed in the cornea (*n* = 1 of 22, marked with arrowhead; Figure 6B, Table 4). Menthol was found to show an unequivocal sensitizing effect only in a minority of fibers with high threshold temperature as outlined in supplement of Zimmermann et al. (2011); in many fibers menthol application caused a decreased response with reduced peak firing rate and increased adaptation with some cold responses being entirely blocked (Zimmermann et al., 2011; Toro et al., 2015). Given the encoding deficit of CC-fibers in TRPM8-deficient mice (Toro et al., 2015), the lack of apparent sensitization is not a lack of effect of menthol, but likely due to excessive depolarization and inactivation of sodium channels.

**Figure 6:** Characteristics of monomodal thermoreceptors (CC-fibers) found in mouse saphenous-nerve of C57BL/6J, TRPM8^−/−^ and DKO. The receptive fields were identified by passing little ice cubes over the skin nerve preparation (see text). **(A)** Averaged histogram summarizing the cold responses of C57BL/6J (gray, *n* = 22), TRPM8^−/−^ (cyan, *n* = 5) and DKO (blue, *n* = 1) in bins of 2 s. Adjacent data points were subjected to 3 pt averaging. Cold responses were reduced in both transgenic strains and representative sample recordings are shown in the right panel for C57BL/6J in black and TRPM8^−/−^ in cyan. The lower traces illustrate the temperature time course. **(B)** Dynamic range of all CC-fibers. Closed squares represent temperature thresholds and closed circles mark temperature of last action potential. Note that most CC-fibers in the mouse regularly encode noxious temperatures with slow adaptation <10°C (one exception marked with arrowhead silenced at 18°C) which often corresponds to the lowest cold ramp temperature indicated in the graph (dashed line and SD as white area). **(C)** The relative frequency of CC-fibers in the saphenous nerve is given as percentage and was estimated by determining the number of split bundles which contained CC-fibers. The search included 54 fine splits in C57BL/6J, and 106 each in TRPM8^−/−^ and DKO. **(D–G)** Quantification of parameters illustrating **(D)** response magnitude counted as action potentials per 60 s cold stimulus, **(E)** peak firing frequency, **(F)** static response quantified as fraction of the action potentials discharged during the constant cold stimulus (16–60 s) and, **(G)** threshold temperatures of activation. All values are given in Table 4. Asterisks refer to Student's *t*-test. Boxes illustrate mean and upper and lower quartiles.

**Table 4:** Properties of cold thermoreceptors in C57BL/6J and 129S1/SvImJ mice.

**Strain**	***n***	**Number of action potentials per 60 s cold stimulus**	**Static cold response as % of entire response**	**Peak DC (1/s)**	**Mean DC (1/s)**	**Threshold temperature** °**C**	**Conduction velocity (m/s)**	**Test with glass rod**	**Measured cold spot density (% per tested fiber bundles)**
							**Mean (min/max)**		
C57BL/6J	22	390.8 ± 193.3	54.8 ± 20.1	64.5 ± 30.7	18.4 ± 11.3	24.3 ± 5.0 (15.5/31.8)	Not determined	All negative	18.5 (10/54; *n* = 3 mice)
129S1/SvImJ	11	382.6 ± 204.9	61.9 ± 30.5	57.1 ± 23.8	18.3 ± 10.1	26.6± 4.1 (21.1/34.9)	0.56 ± 0.43 (0.28/1.76)	All negative	Not determined
TRPM8^−/−^	5	85.0 ± 45.5	31.1 ± 13.8	16.0 ± 6.5	4.9 ± 2.4	31.1 ± 2.0 (28.3/33.7)	Not determined	2 positive	2.8 (3/106; *n* = 4 mice)
DKO TRPM8A1^−/−^	1	88	50	16.6	4.3	21.8	Not determined	Very high threshold	0.9 (1/106; *n* = 7 mice)

*Recordings from 129S1/SvImJ were from a previous study (Zimmermann et al., 2011). In C57BL/6J and TRPM8^−/−^ some recordings were included from a previous publication (Toro et al., 2015); All values are mean ± SD*.

To estimate the relative frequency of these fibers in the saphenous nerve, we counted the number of cold spots (using ice cube test) per thinly split nerve bundle. Cold spots where then isolated with the Teflon ring and systematically evaluated whether they were single fibers (for details see Section Methods). In the C57BL/6J mice, we tested 54 bundles (see Table 4, Figure 6C). In 10, we identified single or multiple unimodal cold spots by slowly passing small ice cubes close to the skin surface. None of them were sensitive to application of high mechanical pressure with the glass rod. In TRPM8^−/−^, we tested 106 bundles in preparations from four mice and found only 3 cold spots. They were all sensitive to mechanical stimulation, but shared more similarity with CC-fiber responses than to the previously described multimodal nociceptors. In DKO mice we tested 106 bundles from seven mice and identified one CC-fiber like response; also this fiber was mechanosensitive, albeit with a very high mechanical threshold. Presumably the relative frequency of cold spots is strongly reduced in the absence of TRPM8 and, TRPA1 may be involved in the encoding of some of the remaining responses. In addition to the reduced incidence, absence of TRPM8 reduced response magnitude, mean, and peak discharge to one-fifth of the average wildtype cold spot response (Figures 6D,E) and further increased adaptation (Figure 6F) and led to a different threshold temperature (Figure 6G).

### TRPM8 function in A-fiber mechanocold nociceptors

The pattern of encoding cold stimulus intensity in murine Aδ-fibers is different from that in C-fiber mechanocold nociceptors and from Aδ-fibers in cats or primates; this makes the significance of this fiber type for cold temperature sensing in the mouse somatosensory system difficult to judge. Cold-sensitive A-fibers in both the C57BL/6J and the 129S1/SvImJ strain are infrequent. In contrast to this appears the fact that stimulation with temperatures below 0°C excites all Aδ-fibers in the rat (Simone and Kajander, 1997). With a stimulus temperature ramp between 30 and 5°C, we found that Aδ-fibers have smaller cold responses, lower peak and mean firing rates as compared to the C-fibers and menthol has an almost negligible sensitizing effect. Aδ-fiber cold responses also cover a variable range of thresholds (Table 5). In addition, while cold responses in C-fibers nociceptors are steady and reproducible (Zimmermann et al., 2009; Vetter et al., 2013), in A-fibers repeatedly applied cold stimuli in intervals of 3–5 min do often create highly variable responses or are not reproducible. In Table 5, the encoding properties are therefore enlisted as average of two consecutive cold stimuli. In our C57BL/6J sample of 47 A-fibers, 25% (*n* = 12) of the fibers responded to cold, but only 2 (17%) showed sensitization in response to 100 μM menthol, i.e., increased their cold response or peak discharge rate after application of menthol. Menthol may also act through TRPA1 and a desensitizing effect due to depolarization shunt may also be a sign of TRPM8 or TRPA1 expression, but the small responses and the lack of reproducibility, make it difficult to investigate molecular mechanisms. Nevertheless, in the 129S1/SvImJ strain a similar small fraction of cold responses were sensitized by 500 μM menthol (13%) and the A-fibers had similar properties (Table 5). Because of these difficulties, we did not search for this type of cold nociceptor in the knockout strains.

**Table 5:** Properties of cold-sensitive A-fibers in C57BL/6J and 129S1/SvImJ mice.

**Strain**	**Fiber type**	**Frequency and pharmacology of TRPM8 status (**+**/**−**)**			**Number of Action potential per 60 s cold stimulus**^b^	**Peak DC of cold response (1/s)**^b^	**Mean DC of cold response (1/s)**^b^	**Thresh. temp. of cold response (°C)**^b^	**Conduction Velocity (m/s)**	**von Frey threshold (mN)**
								**Mean (min/max)**	**Mean (min/max)**	**Median (min/max)**
C57BL/6J *n* = 47	AM	35 (75%)	+	3 (8.6%)^a^	9.0 ± 7.0	1.8 ± 1.1	0.6 ± 0.3	19.4 ± 2.4	3.3 ± 1.9 (1.8/5.5)	4.0 (4/4)
			−	32 (91.4%)	−	−	−	–	8.4 ± 3.6 (1.1/13.6)	4.85 (1/22.6)
	AMC	12 (25%)	+	2 (17%)	1.5 ± 0.0	0.02 ± 0.0	0.01 ± 0.0	15.6 ± 6.7 (9.4/29.6)	5.5 ± 4.2 (2.5/8.4)	3.4 (2.8/4)
			−	10 (83%)	5.3 ± 4.6	1.6 ± 1.4	0.6 ± 0.5	15.8 ± 5.6 (6.6/24.8)	8.0 ± 2.7 (6.5 /11.8)	4.9 (2/16)
129S1/SvImJ *n* = 65	AM	50 (77%)	+	3 (6%)^a^	12.3 ± 2.3	33.2 ± 38.2	4.4 ± 4.1	26.2 ± 1.5 (25.1/27.2)	8.7 ± 3.0 (5.2/10.7)	1.0 (1/16)
			−	47 (94%)	−	−	−	–	7.6 ± 3.6 (1.6/15.8)	1.0 (1/16)
	AMC	15 (23%)	+	2 (13%)	10.0 ± 9.9	2.7 ± 3.4	0.5 ± 0.5	26.6 ± 4.3 (23.6/29.6)	8.3 ± 9.7 (1.5/15.2)	4.3 (2.8/5.7)
			−	13 (87%)	10.1 ± 9.4	15.5 ± 31.4^*^	4.3 ± 8.0	21.3 ± 7.8 (6.8/30.9)	7.2 ± 3.7 (1.4/13.4)	1.0 (1/45)

*Recordings from 129S1/SvImJ were from a previous study (Zimmermann et al., 2011)*.

a *new cold response after menthol 500 μM (129S1/SvImJ) or 100 μM (C57BL/6J)*;

b *Calculated from the mean of two consecutive cold stimuli; All values are mean ± SD*.

## Discussion

Our results illustrate that both TRPM8 and TRPA1 are required for the detection of environmental cool and noxious cold and seem to represent complementary or synergistic cold transduction systems. From our behavioral findings, it appears that the acute cold avoidance still observed in TRPM8^−/−^ in the temperature range between 28 and 15°C is contributed by the function of TRPA1, because DKO behaved indifferent from random behavior. This early behavior is clearly different from late behavior in the gradient and therefore more likely to be correlated with sensory afferent activity. In the past TRPA1's contribution to cold avoidance was underestimated, because it became only apparent in nocifensive assays, especially cold plate and tail withdrawal, with results being divergent in the literature (Kwan et al., 2006; Karashima et al., 2009; Gentry et al., 2010; Pogorzala et al., 2013). TRPA1 function in cold sensing is probably less ostensible, because our findings pointed out that it acts as cold transducer in a proportion of the TRPM8-deficient cold nociceptor fibers which produce smaller responses, fire at lower rates, and are more prone to adaptation upon constant cold stimulation than the dominant TRPM8-expressing cold nociceptor and thermoreceptor types. A recent study using the *ex vivo* somatosensory system preparation investigated the difference in cold-activated firing in TRPM8-positive and negative neurons and confirmed peak instantaneous frequency to be highest in TRPM8-positive neurons (Jankowski et al., 2017).

More complex behavioral setups, such as the 2TC assay, our thermal gradient ring or the elongated form of the thermal gradient test integrate multiple level information including primary afferent detection, spinal cord processing and brain processes of perception, decision making, and thermoregulation (Touska et al., 2016). In this sense, we already found a remarkable speeding of warm seeking behavior in the 15–40°C ring track (Touska et al., 2016) and we confirmed here that in the 5–30°C environment, TRPA1^−/−^ have a remarkable lack of early and late locomotive behavior in the cold zones <13°C which may be due to a wiring of TRPA1-pathways to warm-sensing pathways in the spinal cord similar to other observations (McCoy et al., 2013) or have to do with TRPA1 being also active as heat sensor (Moparthi et al., 2014; Yarmolinsky et al., 2016).

We observed that TRPM8 empowers cold nociceptors to produce sustained cold responses in nociceptors and that it is largely required to encode graded cold stimuli in the unimodal thermoreceptors (Zimmermann et al., 2011; Toro et al., 2015) and we also found that these two features are apparently not or only little compensated when TRPM8 is lost. Therefore, TRPA1's distinctive contribution to cold avoidance behavior must necessarily become more apparent in the absence of TRPM8 and, on the other hand, the lack of cold transduction by TRPA1 is in large parts compensated by the dominant and powerful TRPM8 transducer. When estimated from our recordings, cold nociceptors deficient of TRPM8 produce one quarter or one-fifth (depending on the strain) of the response of TRPM8+ nociceptors, but they activate at 5°C higher thresholds and they represent the larger proportion of the cold nociceptors (~60% in both strains). The distinct features of this fiber class may therefore be able to compensate well for lack of TRPM8 in the larger ring environment with the higher thermal resolution, but they are apparently less efficient in the smaller ring environment with the steeper gradient (Touska et al., 2016).

The resistance of TRPM8+ nociceptor cold responses to adaptation appears quite striking. It is likely that this is not a feature of the TRPM8 receptor alone, although it is known that a number of cellular signaling pathways including presence of phosphatidylinositol 4,5-bisphosphate and reduced activity of phospholipase C (Yudin et al., 2011, 2016) sensitize TRPM8 to produce larger currents *in vitro*, it is also likely that TRPM8 activation triggers secondary responses, such as the closure of the panneuronal M-channels which lead to substantial increase in the static response of the cold nociceptors (Vetter et al., 2013).

The DKO mice have remarkably larger cold avoidance deficits than TRPM8^−/−^ and this even affected their preferred temperature range at the end of the 60 min measurement where they show a largely erratic behavior. Although, DKO act randomly in the first 15 min in the ring track adjusted to 15–40°C, where other strains already show distinctive cold avoidance, cold avoidance is still not extinguished in this strain. When noxious cold temperatures are included and ring temperatures lowered to 5–30°C, clear cold avoidance—although much less than in any other strain—became apparent. The DKO do also still judge warmer areas as preferable during late observation periods which may account for other cold transduction mechanisms of which for example KCNK potassium channels are identified and act synergistic to the cooling-induced excitability increase (Zimmermann et al., 2007; Noel et al., 2009; Palkar et al., 2015) or the recent suggestion of a Na_V_1.9 carrying fiber population with separate transduction mechanism (Lolignier et al., 2015) could be a match. The delayed onset of cold avoidance in DKO is explained by the large lack of two populations of cold nociceptors and the largest part of the unimodal cold thermoreceptors. Nevertheless, DKO cold nociceptors are still able to produce large cold responses although they are scarce and appeared as outlier in our fiber survey, they are apparently sufficient to mediate slow onset cold avoidance to noxious temperatures.

In part our results are in conflict with results from a 2TC assay and with measurement of c-fos expression that identified DKO as indifferent from TRPM8^−/−^ (Knowlton et al., 2010). We previously found evidence with fMRI measurements in TRPA1-deficient mice that support TRPA1-mediated cold temperature detection at 15°C (Vetter et al., 2012). These conclusions are supported by the present findings in the thermal running track, where DKO, but not TRPA1^−/−^ or TRPM8^−/−^, move randomly (in the 15–40°C gradient) for the temperatures between 27 and 15°C during the early exploratory phase. Nevertheless, cold avoidance does evolve over time in DKO and becomes apparent in the final 15 min of the measurement and much more pronounced with inclusion of noxious temperatures. We believe that the circular gradient assay does provide a more accurate measure of cold avoidance and preference behavior, as it enforces locomotion in mice. This setup also enforces the repeated exposure to cold temperature as the absence of corners or semi separating walls does not restrict movements or provoke counterproductive idleness (Dhaka et al., 2007; Touska et al., 2016). In our setup, it is therefore likely that the mice do avoid cold deliberately and specifically, unless they lack either the ability to perceive cold or the ability to learn to avoid it, which means that memory deficits should affect the cold avoidance readout in later time bins. Although, TRPA1 channels where recently shown to be involved in hippocampal long-term potentiation (Shigetomi et al., 2013), it is likely that this did not affect the cold avoidance measure, because the TRPA1^−/−^ acted like the matched C57BL/6J control and DKO still did show a significant evolution of its reduced cold avoidance phenotype at later time points.

Surprisingly, in contrast to previous measurements in the 2TC assays (Bautista et al., 2007; Dhaka et al., 2007), the cold avoidance deficit of TRPM8^−/−^ is relatively small in the 5–30°C gradient assay, and is apparent only in a broader early and late distribution in the 12-zone histogram for the warmest three zones, which is in accordance with the findings in the 15–40°C environment, where we also identified a broader distribution in the late bins. This is also visible in the cumulative response functions for both temperature ranges. Nevertheless, the huge cold avoidance deficit of the TRPM8^−/−^ in the small ring with the lower resolution (Touska et al., 2016) implies that cold temperature encoding integrates many different factors including the stimulus characteristics, differential afferent activity and activation of different cold pain pathways and their wiring in the spinal cord.

## Author contributions

ZW, PG, SE, and KZ performed experiment and analyzed data. FT analyzed data and calculated statistics. ZW, PG, FT, and KZ wrote the manuscript.

### Conflict of interest statement

The authors declare that the research was conducted in the absence of any commercial or financial relationships that could be construed as a potential conflict of interest.
